The article "The Efficacy of Repetitive Transorbital Alternating Current Stimulation (rtACS) in Patients With Optic Nerve Damage: A Systematic Review and Meta-Analysis" was published in 2024. Journal: Cureus.

# The Efficacy of Repetitive Transorbital Alternating Current Stimulation (rtACS) in Patients With Optic Nerve Damage: A Systematic Review and Meta-Analysis

**DOI:** 10.7759/cureus.76669

**Published:** 2024-12-31

**Authors:** Ali S Alsudais, Ziad M Bukhari, Talal Alajmi, Manar M Alamri, Fay Alsuhaym, Ahad Alotaibi, Lama B Alharbi, Atheer Aboud, Basil K Alshammari, Ahmad Aljumaah, Ismail Tuwir

**Affiliations:** 1 College of Medicine, King Saud Bin Abdulaziz University, Jeddah, SAU; 2 Department of Ophthalmology, King Abdulaziz Medical City, Ministry of National Guard Health Affairs, Jeddah, SAU; 3 College of Medicine, King Saud Bin Abdulaziz University for Health Sciences College of Medicine, Jeddah, SAU; 4 Faculty of Medicine, King Khalid University, Abha, SAU; 5 College of Medicine, Princess Nourah bint Abdulrahman University, Riyadh, SAU; 6 College of Medicine, University of Jeddah, Jeddah, SAU; 7 College of Medicine and Medical Science, Arabian Gulf University, Manama, BHR; 8 College of Medicine, Jouf University, Aljouf, SAU; 9 College of Medicine, Royal College of Surgeons in Ireland, Riyadh, SAU

**Keywords:** alternating current stimulation, optic neuropathy, rtacs, vision restoration, visual field

## Abstract

Optic nerve disorders significantly contribute to visual impairment with irreversible visual deficits. Current treatments have limited efficacy in resolving chronic visual deficits, necessitating novel therapeutic strategies. Neurorehabilitation techniques, including repetitive transorbital alternating current stimulation (rtACS), have emerged as promising approaches to restore lost visual function through the ability to modulate brain activity. However, the evidence on the effectiveness of rtACS remains inconclusive, warranting a systematic review to assess its potential as a therapeutic intervention for optic nerve-related visual deficits. This study exclusively evaluated the effectiveness of rtACS for visual field restoration in patients with optic nerve damage, including only randomized controlled trials (RCTs) that met the strict eligibility criteria. A thorough screening and data extraction process was conducted by independent reviewers, followed by a meta-analysis to assess the statistical significance and heterogeneity of the included studies. The improvement in the visual field in the rtACS compared to the sham group was the primary outcome, and visual acuity improvement was the secondary outcome. This study included three RCTs that evaluated the effects of rtACS compared to sham control in treating optic nerve damage. In regard to visual field (VF), the results revealed a significant improvement in the detection accuracy of the rtACS group compared to the control group, with a pooled mean difference of 32.06 [95% CI: 19.2, 51.2] (p=0.001, I2= 0%). The near and far vision revealed no statistically significant difference between both groups. Based on the systematic review, the use of rtACS shows a promising effect in improving the detection accuracy of the VF for patients with optic nerve damage, with a significant benefit over sham control. However, the effects on other visual outcomes were minimal, and safety data was limited. Further high-quality trials are needed to corroborate the findings and provide a more comprehensive evaluation of its efficacy and safety for treating optic nerve-related visual deficits.

## Introduction and background

Optic nerve disorders constitute a significant public health concern, contributing substantially to visual impairment and disability worldwide [1]. These disorders, encompassing a spectrum of pathologies including inflammation, ischemia, trauma, and genetic predisposition, can lead to a range of debilitating visual impairments, including color perception deficits, reduced visual acuity, and characteristic visual field defects [2]. The irreversible nature of these visual field defects, often resulting from damage to the optic nerve or visual cortex, poses a significant challenge for the patients, severely impacting their daily activities and diminishing their vision-related quality of life (VRQoL) [3,4].

Current therapeutic interventions for optic neuropathy, such as optic canal decompression surgery and corticosteroid therapy, have demonstrated limited efficacy in completely resolving chronic visual deficits [3]. This unmet clinical need underscores the urgent requirement for novel therapeutic strategies, particularly for patients in the chronic stage of optic neuropathy [3].

In recent years, a burgeoning field of neurorehabilitation techniques has emerged, aiming to activate residual visual pathways and potentially restore lost visual function [5]. These techniques, including behavioral vision training, vision restoration therapy, and transorbital low-intensity electrical stimulation (TES), hold promise for improving visual function in individuals with optic nerve damage [5]. Among these approaches, transorbital alternating current stimulation (tACS), a form of TES, has garnered considerable attention due to its potential to modulate oscillatory brain activity through the entrainment of specific stimulation frequencies [6,7].

While tACS, particularly in its repetitive form (rtACS), has shown promise in enhancing visual performance following optic nerve damage, the evidence remains inconclusive due to the limited sample sizes in most studies [8-10]. Therefore, a systematic and critical review of the available literature on the effectiveness of rtACS in visual field restoration for patients with optic nerve damage is warranted to assess the potential of this emerging therapeutic modality. This review will critically evaluate the existing evidence base, identify knowledge gaps, and provide recommendations for future research directions.

## Review

Methodology

This study was a systematic review and meta-analysis that closely followed the established PRISMA (Preferred Reporting Items for Systematic Reviews and Meta-Analyses) guidelines throughout its planning, execution, and reporting processes [11]. Additionally, the researchers registered the study protocol prospectively in the PROSPERO (International Prospective Register of Systematic Reviews) database, which was assigned the identifier [CRD42023457913].

This study exclusively included only randomized controlled trials (RCTs) about rtACS efficacy in visual field restoration in optic neuropathy with residual vision and stable visual field loss. We excluded reviews, articles written in languages other than English, non-RCTs, and studies using any other electrical stimulation modality other than rtACS studies. The primary outcome of this review was comparing the changes noticed in the areas of visual field loss between the rtACS and control groups. These changes were measured as a percentage called detection accuracy (DA). DA will compare the change of VF to the baseline. Other secondary outcomes evaluated in our review included visual acuity at near and far distances and any adverse event of rtACS.

A systematic review search was performed to cover all published studies from inception without language or national limitations. The search was performed in August 2023 in the following medical databases that were searched: PubMed, Central, Scopus, DOAJ, and CTG. The data search strategy included these terms: “optic nerve damage,” “optic neuropathy,” ischemic optic neuropathy,” “visual field,” “vision,” ”VF,” “visual field restoration,” “vision restoration,” “noninvasive repetitive transorbital alternating current stimulation,” “repetitive transorbital alternating current stimulation,” “transorbital alternating current stimulation,” “transorbital stimulation,” “alternating current stimulation,” “transorbital alternating,” “transorbital,” and “rtACS.” Also, the reference lists of included articles were manually reviewed to identify any more relevant articles.

Independently and in pairs, two reviewers complied with the eligibility criteria and performed title and abstract screening, full-text assessment, and data extraction from the included RCTs. Discrepancies were discussed with a third reviewer or resolved through consensus before further advancement. Data were extracted in Microsoft Office Excel (Redmond, USA) using a predefined template. The extracted data included the following information: authors, year of publication, study design, study population, country, control group, number of patients, number of eyes, electrode type, position of active/reference electrode, frequency (Hz), pulse period, electrical stimulation (ES) parameters current strength, session duration, treatment frequency (number of ES sessions), condition, measured outcomes, exclusion criteria, and conclusion.

The quality of evidence for each outcome was assessed independently, and together, two reviewers used the Cochrane Risk of Bias 2 (RoB2) tool to assess the risk of bias in the eligible RCTs [12]. Each study's risk of bias was reviewed and categorized as high, low, or some concerns. Discrepancies between the reviewers were resolved through discussion until an agreement was reached.

Data analysis was performed using RevMan (Review Manager) version 5.3 (Cochrane Collaboration). The meta-analysis was performed using the random-effects model. A 95% confidence level and p < 0.05 were set for statistical significance. The statistical heterogeneity was assessed using the I2.

Results

Our systematic review began with 1,140 records identified from databases and registries (Figure 1). After the initial screening, we excluded 1,118 records mainly due to their irrelevance. Although we aimed to retrieve 22 full reports, 10 of them were not available. After evaluating the eligibility of the remaining 12 reports, we excluded nine of them: two for utilizing concurrent brain stimulation modalities and seven for reporting different outcomes. In the end, our review included three RCTs that met our inclusion criteria [3,13,14].

**Figure 1:** : PRISMA flowchart

Two independent reviewers, namely A.A. and Z.B., systematically employed the RoB 2 tool to individually appraise the potential sources of bias in the eligible RCTs [12]. Any discrepancy was solved by agreement between reviewers. Two of the three trials in this investigation exhibited a low risk of bias, and one trial had some concerns regarding the risk of bias as visually depicted in Figure 2.

**Figure 2:** Risk of bias assessment of the included studies D1: Randomization process; D2: Deviations from the intended interventions; D3: Missing outcome data; D4: Measurement of the outcome; D5: Selection of the reported result

Our study included three RCTs conducted in Germany examining the effects of taACS compared to a vehicle/sham in treating optic nerve damage [3,13,14]. The mean ages ranged from 52.3 to 57.8 years in the tACS groups and 51.9 to 62.9 years in the vehicle groups, with standard deviations generally around 14-15 years. The studies were published in 2011 and 2016, as shown in Table 1.

**Table 1:** Characteristics of included studies rtACS: Repetitive transorbital alternating current stimulation

Authors	Country	Number of participants (eyes)		Age in years (Mean±Standard Deviations)	
		tACS	Vehicle	tACS	Vehicle
Gall C et. al. 2011 [3]	Germany	24 (40)	18 (30)	52.7±15.7	62.9 ±7.0
Gall C et. al. 2016 [13]	Germany	45	37	57.8 ± 14.2	60.7 ± 11.6
Sabel BA et. al. 2011 [14]	Germany	12 (24 eyes)	10 (20)	52.3±14.3	51.9±17.3

Our meta-analysis examined the detection accuracy as the primary outcome by combining data from three RCTs. The results revealed a significant improvement in the treatment group compared to the control group, with a pooled mean difference of 32.06 [95% CI: 19.2, 51.2]. The analysis showed a significant p-value and no heterogeneity (p=0.001, I2= 0%), indicating a strong and consistent effect (Figure 3).

**Figure 3:** Forest plot of detection accuracy Gall C. et al. 2016 [13]; Gall C. et al. 2011 [3]; Sabel BA. et al. 2016 [14]

Additionally, two of the three RCTs [13,14] have counted change in near and far vision as one of the secondary outcome measures. The result of both outcomes revealed a minimal pooled mean difference in favor of tACS over sham control, with an effect size of 0.02 for both outcomes. For near vision change, this difference fell within a 95% confidence interval of (0.03, 0.07), though it was not statistically significant with no substantial heterogeneity (p=0.50, I2=0%). Similarly, far vision change showed a mean difference of 0.02 within a 95% confidence interval of (0.03, 0.08), also without reaching statistical significance with no substantial heterogeneity (p=0.39, I2= 0%) (Figures 4, 5).

**Figure 4:** Forest plot of near vision Gall C. et al. 2016 [13]; Sabel BA. et al. 2016 [14]

**Figure 5:** Forest plot of far vision Gall C. et al. 2016 [13]; Sabel BA. et al. 2016 [14]

Except for the study conducted by Gall C. et al. (2016) [13], there was insufficient data available on the safety profile in all the studies. Gall C. et al. reported the occurrence of minor adverse effects such as mild headache, discomfort, vertigo, and mild uncomfortable sensations.

Discussion

Our systematic review aimed to assess the efficacy and safety of rtACS in treating optic nerve damage. Only three studies out of 1,140 records met the inclusion criteria. Our study combined data from three RCTs to examine the accuracy of detection in VF as the primary result.

The results showed a statistically significant improvement and a higher DA in the rtACS group compared to the control group in the VF with optic nerve damage, as highlighted by the lack of heterogeneity (I² = 0%) as shown in Figure 3. In addition, two of the three randomized controlled trials considered changes in near and far vision as secondary outcome measures [13,14]. The results indicated a minimal pooled mean difference favoring rtACS over sham control. The difference in near vision did not reach statistical significance and showed no substantial heterogeneity. Similarly, the change in far vision revealed a lack of statistical significance and exhibited no substantial heterogeneity, as shown in Figures 4, 5.

These improvements could be due to indirect effects mediated by the synchronized activation patterns induced in the retinal ganglion cells [15]. In other words, the hypothesis suggests that rtACS may be able to influence and potentially improve perceptual abilities and sensory thresholds within regions of the visual system that still retain some degree of functional capacity, much like what has been observed with other stimulation approaches [3,9,10,14]. The therapeutic effect of rtACS may be after the process of re-synchronizing the brain network, hence, amplifying the already damaged residual vision [6,16].

Assessing the safety profile of rtACS was one of the main secondary outcomes of our study. Except for the study conducted by Gall C. et al. [13], there was insufficient data available on the safety profile in all the studies. Few adverse events were reported, such as headache, discomfort, vertigo, and mild uncomfortable sensations.

Our study reaffirms and expands upon the findings of Navarro et al. [17] in studying the effectiveness and safety of non-invasive electrical stimulation for vision restoration by narrowing the scope to rtACS and providing a more practical and specific resource for clinical decision-making and patient care in our study. In this study, we address critical nuances and limitations in the current evidence base that may not have been fully explored in the broader meta-analysis by Navarro et al. [17], such as near and far vision. 

Clinically, the findings suggest that rtACS could be considered as an adjunct treatment for patients with optic nerve damage to improve the visual abilities. However, the clinicians should have realistic expectations regarding the extent of visual recovery, as there was a minimal improvement for near and far vision. Furthermore, the lack of substantial safety data limits the ability to fully endorse rtACS without reservations. 

One strength of this review is the accurate selection process, which ensured that only studies meeting inclusion criteria were analyzed, thereby enhancing the reliability of the findings. The use of meta-analysis to pool data from multiple studies also adds robustness to the results. However, several limitations need to be acknowledged. First, the small number of included studies limits the generalizability of the findings. Also, the inability to access 10 potentially relevant full reports may have introduced selection bias. Moreover, the variability in study demographics and the limited geographical focus (all studies conducted in Germany) further restrict the applicability of the findings to broader populations.

Future research should focus on conducting larger, multicentric randomized controlled trials to confirm the efficacy of rtACS in diverse populations. These studies should aim to provide comprehensive data on secondary outcomes, such as near and far vision, and include detailed safety profiles to better understand the potential adverse effects.

## Conclusions

In conclusion, this systematic review provides compelling evidence for the potential of rtACS as an innovative therapeutic intervention for improving the visual field in patients with optic nerve damage. The analysis of the included randomized controlled trials (RCTs) demonstrates a significant advantage of rtACS over sham treatments, indicating its role in the possibility of modulating brain activity to enhance visual function. While the findings reveal marked improvements in the visual field, it is important to note that the effects on visual acuity and other visual outcomes were minimal and did not achieve statistical significance. This discrepancy highlights the complexity of visual rehabilitation and suggests that rtACS may primarily affect specific aspects of visual processing rather than providing a comprehensive solution for all visual deficits. Moreover, the limited safety data available from the reviewed studies calls for a cautious interpretation of the results. As such, further high-quality trials are essential to corroborate these findings and to better understand the long-term effects and safety profile of rtACS. Future research should also explore optimal treatment parameters, including frequency, duration, and patient selection, to maximize therapeutic benefits.

## References

[1] Biousse V, Newman NJ (20161). Diagnosis and clinical features of common optic neuropathies. Lancet Neurology.

[2] Touitou V, LeHoang P (2012). Diagnostic approach in optic neuropathy. Rev Neurol (Paris).

[3] Gall C, Sgorzaly S, Schmidt S, Brandt S, Fedorov A, Sabel BA (2011). Noninvasive transorbital alternating current stimulation improves subjective visual functioning and vision-related quality of life in optic neuropathy. Brain Stimul.

[4] Greenwald BD, Kapoor N, Singh AD (2012). Visual impairments in the first year after traumatic brain injury. Brain Inj.

[5] Sabel BA, Hamid AI, Borrmann C, Speck O, Antal A (2020). Transorbital alternating current stimulation modifies BOLD activity in healthy subjects and in a stroke patient with hemianopia: A 7 Tesla fMRI feasibility study. Int J Psychophysiol.

[6] Sabel BA, Henrich-Noack P, Fedorov A, Gall C (2011). Vision restoration after brain and retina damage: the "residual vision activation theory". Prog Brain Res.

[7] Zaehle T, Rach S, Herrmann CS (2010). Transcranial alternating current stimulation enhances individual alpha activity in human EEG. PLoS One.

[8] Henrich-Noack P, Sergeeva EG, Eber T (2017). Electrical brain stimulation induces dendritic stripping but improves survival of silent neurons after optic nerve damage. Sci Rep.

[9] Bola M, Gall C, Moewes C, Fedorov A, Hinrichs H, Sabel BA (2014). Brain functional connectivity network breakdown and restoration in blindness. Neurology.

[10] Schmidt S, Mante A, Rönnefarth M, Fleischmann R, Gall C, Brandt SA (2013). Progressive enhancement of alpha activity and visual function in patients with optic neuropathy: a two-week repeated session alternating current stimulation study. Brain Stimul.

[11] Page MJ, McKenzie JE, Bossuyt PM (2021). The PRISMA 2020 statement: an updated guideline for reporting systematic reviews. BMJ.

[12] Sterne JA, Savović J, Page MJ (2019). RoB 2: a revised tool for assessing risk of bias in randomised trials. BMJ.

[13] Gall C, Schmidt S, Schittkowski MP (2016). Alternating current stimulation for vision restoration after optic nerve damage: a randomized clinical trial. PLoS One.

[14] Sabel BA, Fedorov AB, Naue N, Borrmann A, Herrmann C, Gall C (2011). Non-invasive alternating current stimulation improves vision in optic neuropathy. Restor Neurol Neurosci.

[15] Foik AT, Kublik E, Sergeeva EG, Tatlisumak T, Rossini PM, Sabel BA, Waleszczyk WJ (2015). Retinal origin of electrically evoked potentials in response to transcorneal alternating current stimulation in the rat. Invest Ophthalmol Vis Sci.

[16] Bola M, Sabel BA (2015). Dynamic reorganization of brain functional networks during cognition. Neuroimage.

[17] Navarro PA, Contreras-Lopez WO, Tello A, Cardenas PL, Vargas MD, Martinez LC, Yepes-Nuñez JJ (2024). Effectiveness and safety of non-invasive neuromodulation for vision restoration: a systematic review and meta-analysis. Neuroophthalmology.

